# Efficacy of Constructing Digital Hybrid Skull-Dentition Images Using an Intraoral Scanner and Cone-Beam Computed Tomography

**DOI:** 10.1155/2022/8221514

**Published:** 2022-03-03

**Authors:** Joo-Hee Lee, Soo-Hwan Byun, Sang-Min Yi, In-Young Park, Byoung-Eun Yang, Hye-Lim Lee

**Affiliations:** ^1^Division of Pediatric Dentistry, Hallym University Sacred Heart Hospital, Anyang 14066, Republic of Korea; ^2^Division of Oral & Maxillofacial Surgery, Hallym University Sacred Heart Hospital, Anyang 14066, Republic of Korea; ^3^Graduate School of Clinical Dentistry, Hallym University, Chuncheon 24252, Republic of Korea; ^4^Institute of Clinical Dentistry, Hallym University, Chuncheon 24252, Republic of Korea; ^5^Division of Orthodontics, Hallym University Sacred Heart Hospital, Anyang 14066, Republic of Korea

## Abstract

Cone-beam computed tomography (CBCT) can distort dentition, and additional imaging is often required. A plaster model to help digitize dental images has been widely used in clinical practice, but there are some inconveniences such as complexity of the process and the risk of damage. The aim of this study was to evaluate the potential for improving dentition imaging with CBCT scans using an intraoral scanner instead of a plaster model. The study used laser model-scanned images of plaster models, imaging from two intraoral scanners, and CBCT images from 20 patients aged 12-18 years. CS 3600 (Carestream Dental, Atlanta, USA) and i700 (Medit, Seoul, Korea) were used as intraoral scanners. The full arch was scanned at once or in three sections using intraoral scanners. The segmented scans were merged to obtain full-arch images. With i700, full-arch images were additionally acquired using its “smart stich” function. The virtual skull-dentition hybrid images obtained from intraoral scanners were superimposed with images obtained using a plaster cast. The difference and distance of coordinate values at each reference point were measured. The average distances from the images obtained with the plaster cast were smaller than 0.39 mm, which is the voxel size of CBCT. Scanning the complete or partial arch using CS 3600 or i700 satisfactorily complemented the CBCT when compared to the plaster model. The virtual skull-dentition hybrid image obtained from intraoral scanners will be clinically useful, especially for patients and surgeons who have difficulty in scanning the complete arch at once.

## 1. Introduction

The utilization of three-dimensional (3D) digital images to create a virtual treatment plan has recently gained popularity in the dental field [1–3]. In particular, cone-beam computed tomography (CBCT) can be used to provide 3D information on a patient's craniomaxillofacial region. Virtual simulations can be used to plan maxillofacial surgery, and computer-aided design/manufacturing technologies can be used to create dental wafers and implant surgery guides [4–7]. However, CBCT images have limitations in providing accurate information for the following two reasons: first, CBCT images are scattered by enamel, restorations, implants, orthodontic devices, etc., resulting in streak artifacts. Second, the X-ray beam, which is a CBCT measurement method, does not always create perfectly uniform images [8–11]. As the teeth are enlarged, distortion of the occlusal surface of the teeth occurs. Therefore, to display accurate information about the dentition in the CBCT image, it is necessary to supplement it with additional dentition imaging. A virtual skull-dentition hybrid image, created by superimposing a dentition image obtained by a model scan of a plaster model with a CBCT image, is a method that has been widely used in clinical practice [12–14].

When compared to laser scanning of plaster casts, utilizing an intraoral scanner (IOS) provides advantages. The IOS is useful because it can obtain a digital model from the patient without having to take a physical impression, and no pouring of plaster is involved. Furthermore, the digital model from the IOS is not susceptible to damage, requires no storage space, and has much fewer time and space limits when collaborating with other departments. In addition, several patients have found intraoral scanning to be more relaxing than traditional impression taking [15, 16]. Using an IOS, the accuracy of imaging a short span involving one tooth, a quadrant, or sextant is generally comparable to that of the traditional impression method [17]. However, although the accuracy of imaging a long span of the complete arch is improving, it remains controversial [18, 19]. Imaging of the complete arch varies in accuracy depending on the operator's scan strategy [20]. The entire arch scan data may be obtained by performing segmented scanning, which is more accurate and less affected by the scan method; the segmented images are then integrated to create imaging of a complete arch. The Medit i700 (Medit, Seoul, Korea), which was released in 2021, features a “smart stitch” ability in its software that allows common parts between various scan pieces to be joined automatically. If segmented scanning has a high enough clinical accuracy, it can be employed extensively without being influenced by the operator's scan technique. The goal of this study was to determine whether scanning the entire or partial arch with an IOS can help supplement CBCT scans.

## 2. Methods

The study participants were 20 patients between 12 and 18 years of age (9 males, 11 females), who visited the Dentistry Department of Hallym University Sacred Heart Hospital. The patients' data collection was approved and implemented by the Institutional Review Board (IRB No. 2020-07-005-001) of Hallym University Sacred Heart Hospital. The number of study subjects was calculated by using G∗power (ver. 3.0.10, Franz Faul. Universitat, Kiel, Germany) using a significance level of *a* = 0.05, 95% power, and an effect size of 0.80. Only patients with complete eruption of the first molar were selected; patients with cleft palate, craniofacial syndrome, or metal artifacts such as orthodontic devices or metal restorations were excluded. Plaster cast impression, intraoral scan, and CBCT scans were all performed within a span of two weeks for each patient. A retrospective study was conducted using the maxillary component of each patient's plaster model, IOS digital imaging, and CBCT scan imaging obtained at the time of admission. After obtaining an alginate impression, the surface of the plaster model made with a dental plaster (Rhombstone White, Ryoka Dental, Mie-Ken, Japan) was scanned with a desktop model scanner (Freedom UHD, DOF, Inc., Seoul, Korea), and the Surface Tessellation Language (STL) format digital images were acquired. CS 3600 (Carestream Dental, Atlanta, USA) and i700 (Medit, Seoul, Korea) were the intraoral scanners used. For each patient, the same clinician (JH Lee) performed an intraoral scan according to the manufacturer's instructions to acquire digital images in STL format. CBCT was performed using Alphard 3030 (Asahi, Inc., Kyoto, Japan) with a Frankfort plane parallel to the horizontal plane, field of view 200 × 200 mm, voxel size 0.39 mm, exposure conditions 80 kVP, 5 mA, and 17 s. CBCT images were converted to Digital Imaging and Communications in Medicine (DICOM) format and reconstructed three-dimensionally. Using an IOS, the full arch was scanned simultaneously or divided into sectioned scans. When using the CS 3600, the orthodontic mode was used for scanning the full arch, and the prosthetic mode was used for segmented scanning. The i700 did not have separate modes for full arch and segmented scanning. Additional data were obtained using the i700 “smart stich” function; partial scans were obtained, and the program automatically merged the partial scans to create full-dentition data. For segmented scanning, three divisions were made with the following landmarks: the distal half of the right canine to the distal surface of the right rearmost tooth, the mesial half of the right first premolar to the mesial half of the left first premolar, and the distal half of the left canine to the distal surface of the left rearmost tooth. Subsequently, each divided scanned image was semiautomatically merged based on the overlapping scan images using Geomagic Freeform Plus (3D Systems) to obtain a full-arch dental scan image (STL). Accordingly, six dentition images were obtained from each patient. The CBCT image (DICOM) and each dentition scan image (STL) were transmitted to R2GATE™ (MegaGen Implant Co., Ltd.). Semiautomatic merging was performed based on the midpoint of the incisal edge of the maxillary left and right central incisors and the mesiobuccal cusp of the maxillary left and right first molars. The final virtual skull-dentition hybrid image was obtained by allowing the anatomical head position to be checked from various directions (Figure 1).

Six virtual skull-dentition hybrid image groups per patient were generated:

1. Control group: dentition image obtained by a model scan of plaster cast+CBCT scan
2. Group I: dentition image obtained by scanning the full arch with CS 3600+CBCT scan
3. Group II: dentition image obtained after segmentation scan with CS 3600+CBCT scan
4. Group III: dentition image obtained by scanning the full arch with i700+CBCT scan
5. Group IV: dentition image obtained after segmentation scan with i700+CBCT scan
6. Group V: dentition image obtained after segmentation scan with “smart stitch” function of i700+CBCT scan

In the virtual skull-dentition hybrid image of each group, six anatomical reference points were set and evaluated: the cusp of both canines, the lowest point of the gingival margin of both canines, and the mesiobuccal cusp of both first molars. The three-dimensional information of each reference point was expressed as *x*, *y*, and *z* coordinate values and entered into a program (Geomagic Freeform Plus, 3D Systems, North Carolina, USA). The *x*-axis showed the left-right direction, the *y*-axis showed the up-down direction, and the *z*-axis showed the relationship in the front-back direction. The difference between the coordinate values at each reference point and the distance between the coordinates were measured by superimposing the digital models of the control group and other groups (Figures 2 and 3). Statistical comparisons were made by performing one-way ANOVA and Tukey post hoc tests on the coordinate values and the distance between the coordinates, respectively. Statistical analysis was performed using the Statistical Package for the Social Sciences (SPSS, version 25.0, IBM).

## 3. Results

The mean and standard deviation of each reference point is presented in the tables in this section. The control group is not represented in the table because all values were 0. Except for the *x*-value of the maxillary left canine cusp, statistical analysis indicated significant differences between the groups. To investigate these discrepancies, a post hoc analysis was performed.

Except for two values (the *x*-value of the cusp of the left maxillary canines and the *z*-value of the mesiobuccal cusp of the left first molars), the mean values of group I were significantly different from those of the control group. On the other hand, except for three values (the distance at the mesiobuccal cusp of the maxillary right first molars, *y*-value of the gingival margin's lowest point of the maxillary left canines, and *y*-value of the cusp of the maxillary left canines), the mean values of group II were not significantly different from those of the control group. In general, groups III, IV, and V produced comparable results. The mean values were highest in group I and lowest in group II, but they were all less than the 0.39 mm CBCT voxel size (Tables 1–6).

## 4. Discussion

CBCT is an excellent tool to represent a patient's skull, but it can cause distortion of the dentition. The high density of metal restorations, orthodontic appliances, and enamel is the main cause of distortion [8–11]. Additional dentition images from a plaster cast and IOSs were merged into CBCT images to create virtual skull-dentition hybrid images. Errors can occur using IOSs while scanning and processing [21]. Scanning errors are due to a scanning area, the operator's scanning method and skill, and the type of scanner unit [20, 22]. Filter algorithms are to blame for computer processing errors [23, 24].

The control group (a laser model scanning image of a plaster cast) was compared to the five groups acquired by scanning the complete or partial arch with IOSs. Six different reference points on the virtual skull-dentition hybrid images were compared. In terms of coordinates and distance, the segmented scan using the CS 3600 performed best. When employing the full-arch scan method, segmented scan method, and “smart stitch” feature on the i700, comparable results were obtained. All the results of the i700 showed better outcome than the CS 3600 full-arch scan. Although the mean values of group I of the CS 3600 full-arch scan were significantly different from those of the control group, they were all less than the CBCT voxel size of 0.39 mm. The maximum distance was -0.105 mm in group I at the mesiobuccal cusp of the maxillary right first molars.

The “smart stitch” function in i700 puts partially scanned images together. There will be more errors when more scan image stitching is needed [22]. The function does not require more stitching than the full-arch scan method, but it just changes the order of stitching. When comparing the device CS 3600 and the i700, the i700 is lighter in weight, which could explain why the findings are constant regardless of the scanning method. The i700 weighs 245 g versus 325 g for the CS 3600. The i700 scans twice as fast as the i500, Medit's previous scanner, which scans about twice as fast as the CS 3600.

Baan et al. used a structured light scanner as the gold standard to scan a dried cranium [25]. However, the present study involved real patients, and a control group was created using a virtual skull-dentition hybrid image created using a plaster model. When utilized for orthognathic surgery, this type of hybrid image represented the patient's true dentition in a clinically acceptable manner and displayed the desired surgical result without difficulties [26–31]. Despite the likelihood of errors in merging split-scan images, the split-scan method exhibited improved clinical accuracy when CS 3600 was utilized. When aligning the reference point, a study using the same program as this study found a movement error of 139 *μ*m and an angle error of 2.52 degrees [32]. Variations in accuracy may occur in the process of fusing the CBCT image and the dental image apart from the accuracy of the dental image. Uechi et al. found a root mean square error of 0.4 mm in their study [27]. Gateno et al. found that the error ranged from 0.10 to 0.50 mm [13], while de Waard et al. found that the error ranged from 0.12 to 0.45 mm [33].

It is sometimes required to scan only a portion of the dentition rather than the full dentition simultaneously. A fracture line may extend to the teeth in patients who have fractures in the craniofacial region. In this situation, the data needed for surgery can be collected by scanning each section independently, using the fracture line as a reference, and completing a full-arch image. Patients, including children, who have difficulties opening their mouths for extended periods of time, will feel more at ease with a segmented approach. Furthermore, even for operators who are unfamiliar with intraoral scanning, the segmented scanning method will be useful. The extra step of using another program to merge each segmented scan image is time-consuming and difficult. The i700's “smart stitch” feature can make this step obsolete. This is expected to be a beneficial function, as it will merge scan fragments that were split at the time of scanning if there was a common element between them.

One of the limitations of this study was that it only included participants who did not have orthodontic equipment that could distort the CBCT scan. When a patient is receiving orthodontic treatment, a CBCT scan is obtained to assess the progress of the treatment, or maxillofacial surgery is often performed, and a CBCT scan may be of use. Therefore, more research into the effects of orthodontic equipment, such as brackets, is required. Second, the number of patients involved in this study is insufficient; a larger sample size is needed in future studies to support our findings.

## 5. Conclusion

Scanning the complete or partial arch using CS 3600 or i700 satisfactorily complements the CBCT when compared to the plaster model. A partial arch scan with CS 3600 represented the best results, followed by complete arch scan, partial arch scan, and “smart stitch” function with and full arch scan with CS 3600. This technique shall be widely used clinically for patients and surgeons who find it difficult to scan the complete arch at once, as it can accurately create a virtual skull-dentition hybrid image using an intraoral scanner.

## Figures and Tables

**Figure 1:** Flow charts of the obtaining process of virtual skull-dentition hybrid images of each group.

**Figure 2:** Coordinate value difference and distance between reference points after superimposing the control group and group I.

**Figure 3:** Coordinate value difference and distance between reference points after superimposing the control group and group II.

**Table 1:** Statistical analysis of the coordinate value difference and distance of each group at the lowest point of the gingival margin of maxillary right canines.

		Δ*x*	Δ*y*	Δ*z*	Distance (mm)
I	Average	0.060	0.044	-0.050	-0.078
	SD	0.061	0.061	0.041	0.066
II	Average	0.002	0.004	-0.001	-0.003
	SD	0.017	0.022	0.015	0.026
III	Average	0.009	0.009	-0.002	0.018
	SD	0.027	0.046	0.023	0.056
IV	Average	-0.006	-0.013	-0.002	-0.013
	SD	0.026	0.041	0.012	0.050
V	Average	-0.006	-0.011	0.011	-0.011
	SD	0.026	0.031	0.020	0.047
*F*		12.683	5.805	18.869	10.220
*p* ^1^		0.000^∗^	0.000^∗^	0.000^∗^	0.000^∗^
*T* ^2^		I > III, II, C, V, IV	I > III	V, C, II, IV, III > I	III, C, II, V, IV > I
			III > II, C, V, IV		

^1^Statistical significances were tested by one-way ANOVA among groups (^∗^*p* < 0.05). ^2^Adjustment for multiple comparisons: Tukey.

**Table 2:** Statistical analysis of the coordinate value difference and distance of each group at the cusp of maxillary right canines.

		Δ*x*	Δ*y*	Δ*z*	Distance (mm)
I	Average	0.016	0.061	-0.023	-0.053
	SD	0.017	0.047	0.017	0.039
II	Average	0.000	-0.002	0.001	0.002
	SD	0.008	0.030	0.009	0.024
III	Average	-0.010	-0.003	0.031	-0.042
	SD	0.012	0.025	0.019	0.021
IV	Average	-0.018	-0.008	0.028	-0.040
	SD	0.017	0.021	0.017	0.023
V	Average	-0.017	-0.006	0.035	-0.048
	SD	0.018	0.023	0.019	0.022
*F*		17.608	18.242	44.523	20.272
*p* ^1^		0.000^∗^	0.000^∗^	0.000^∗^	0.000^∗^
*T* ^2^		I > C, II, III	I > C, II, III, V, IV	V, III, IV > II, C > I	II, C > IV, III, V, I
		III > V, IV			

^1^Statistical significances were tested by one-way ANOVA among groups (^∗^*p* < 0.05). ^2^Adjustment for multiple comparisons: Tukey.

**Table 3:** Statistical analysis of the coordinate value difference and distance of each group at the mesiobuccal cusp of maxillary right first molars.

		Δ*x*	Δ*y*	Δ*z*	Distance (mm)
I	Average	0.070	0.145	0.014	-0.105
	SD	0.058	0.098	0.038	0.078
II	Average	0.006	0.015	0.000	-0.011
	SD	0.008	0.024	0.006	0.016
III	Average	-0.006	-0.004	0.039	-0.045
	SD	0.017	0.015	0.016	0.018
IV	Average	-0.005	-0.002	0.031	-0.033
	SD	0.009	0.008	0.015	0.015
V	Average	-0.006	0.001	0.038	-0.043
	SD	0.012	0.017	0.018	0.020
*F*		26.945	38.953	16.950	22.429
*p* ^1^		0.000^∗^	0.000^∗^	0.000^∗^	0.000^∗^
*T* ^2^		I > II, C, IV, V, III	I > II, V, C, IV, III	III, V > IV	C > II
				IV > I	II > IV, V
				I > II, C	IV, V, III > I

^1^Statistical significances were tested by one-way ANOVA among groups (^∗^*p* < 0.05). ^2^Adjustment for multiple comparisons: Tukey.

**Table 4:** Statistical analysis of the coordinate value difference and distance of each group at the lowest point of the gingival margin of maxillary left canines.

		Δ*x*	Δ*y*	Δ*z*	Distance (mm)
I	Average	-0.049	0.023	-0.035	-0.054
	SD	0.044	0.040	0.031	0.048
II	Average	0.013	-0.007	0.011	0.016
	SD	0.034	0.037	0.023	0.044
III	Average	0.000	-0.002	0.005	-0.008
	SD	0.017	0.017	0.015	0.028
IV	Average	0.004	-0.008	0.001	-0.011
	SD	0.019	0.025	0.017	0.035
V	Average	-0.002	0.004	-0.002	0.004
	SD	0.030	0.030	0.027	0.050
*F*		12.620	3.224	11.545	8.084
*p* ^1^		0.000^∗^	0.009^∗^	0.000^∗^	0.000^∗^
*T* ^2^		II, IV, C, III, V > I	I > V, C, III	II, III, IV, C, V > I	II, IV, C, III, V > I
			V, C, III > II, IV		

^1^Statistical significances were tested by one-way ANOVA among groups (^∗^*p* < 0.05). ^2^Adjustment for multiple comparisons: Tukey.

**Table 5:** Statistical analysis of the coordinate value difference and distance of each group at the cusp of maxillary left canines.

		Δ*x*	Δ*y*	Δ*z*	Distance (mm)
I	Average	-0.008	0.033	-0.009	-0.027
	SD	0.014	0.038	0.015	0.030
II	Average	0.001	0.006	-0.001	-0.004
	SD	0.005	0.021	0.008	0.017
III	Average	0.013	-0.022	0.029	-0.053
	SD	0.050	0.037	0.032	0.060
IV	Average	0.013	-0.022	0.041	-0.058
	SD	0.045	0.030	0.054	0.069
V	Average	0.016	-0.022	0.038	-0.061
	SD	0.051	0.041	0.037	0.064
*F*		1.506	10.224	10.685	6.580
*p* ^1^		0.193	0.000^∗^	0.000^∗^	0.000^∗^
*T* ^2^			I > II	IV, V, III > C, II, I	C, II > I
			II > C, V, III		I > III, IV, V
			C, V, III > IV		

^1^Statistical significances were tested by one-way ANOVA among groups (^∗^*p* < 0.05). ^2^Adjustment for multiple comparisons: Tukey.

**Table 6:** Statistical analysis of the coordinate value difference and distance of each group at the mesiobuccal cusp of maxillary left first molars.

		Δ*x*	Δ*y*	Δ*z*	Distance (mm)
I	Average	-0.039	0.119	0.001	-0.086
	SD	0.030	0.108	0.027	0.076
II	Average	-0.004	0.010	-0.001	-0.009
	SD	0.006	0.013	0.003	0.010
III	Average	0.006	-0.008	0.036	-0.042
	SD	0.012	0.018	0.011	0.015
IV	Average	0.010	-0.003	0.026	-0.032
	SD	0.019	0.010	0.015	0.021
V	Average	0.004	-0.004	0.036	-0.041
	SD	0.023	0.015	0.018	0.026
*F*		20.108	23.114	28.873	15.212
*p* ^1^		0.000^∗^	0.000^∗^	0.000^∗^	0.000^∗^
*T* ^2^		IV, III, V, C, II > I	I > II, C, IV, V, III	III, V, IV > I, C, II	C, II > IV
					IV > V, III > I

^1^Statistical significances were tested by one-way ANOVA among groups (^∗^*p* < 0.05). ^2^Adjustment for multiple comparisons: Tukey.

## Data Availability

The data that support the findings of this study are available from the corresponding authors upon reasonable request.
